The article "The Role of the Extracellular Matrix Protein Mindin in Airway Response to Environmental Airways Injury" was retracted in 2016. Reasons: results that could not be reproduced; concerns about the data.

# The Role of the Extracellular Matrix Protein Mindin in Airway Response to Environmental Airways Injury

**DOI:** 10.1289/ehp.1003339

**Published:** 2011-06-17

**Authors:** Sarah Frush, Zhuowei Li, Erin N. Potts, Wanglei Du, Jerry P. Eu, Stavros Garantziotis, You-Wen He, W. Michael Foster, John W. Hollingsworth

**Affiliations:** 1 Division of Pulmonary, Allergy, and Critical Care Medicine, Department of Medicine, Duke University, Durham, North Carolina, USA; 2 National Institute of Environmental Health Sciences, National Institutes of Health, Department of Health and Human Services, Research Triangle Park, North Carolina, USA; 3 Department of Immunology, Duke University, Durham, North Carolina, USA

**Keywords:** airway smooth muscle, endotoxin, innate immunity, lipopolysaccharide, LPS, lung, mindin, ozone, Tlr4, toll-like receptor

## Abstract

Background: Our previous work demonstrated that the extracellular matrix protein mindin contributes to allergic airways disease. However, the role of mindin in nonallergic airways disease has not previously been explored.

Objectives: We hypothesized that mindin would contribute to airways disease after inhalation of either lipopolysaccharide (LPS) or ozone.

Methods: We exposed C57BL/6J and mindin-deficient (^–/–^) mice to aerosolized LPS (0.9 μg/m^3^ for 2.5 hr), saline, ozone (1 ppm for 3 hr), or filtered air (FA). All mice were evaluated 4 hr after LPS/saline  exposure or 24 hr after ozone/FA exposure. We characterized the physiological and biological responses by analysis of airway hyperresponsiveness (AHR) with a computer-controlled small-animal ventilator (FlexiVent), inflammatory cellular recruitment, total protein in bronchoalveolar lavage fluid (BALF), proinflammatory cytokine profiling, and *ex vivo* bronchial ring studies.

Results: After inhalation of LPS, mindin^–/–^ mice demonstrated significantly reduced total cell and neutrophil recruitment into the airspace compared with their wild-type counterparts. Mindin^–/–^ mice also exhibited reduced proinflammatory cytokine production and lower AHR to methacholine challenge by FlexiVent. After inhalation of ozone, mice had no detectible differences in cellular inflammation or total BALF protein dependent on mindin. However, mindin^–/–^ mice were protected from increased proinflammatory cytokine production and AHR compared with their C57BL/6J counterparts. After ozone exposure, bronchial rings derived from mindin^–/–^ mice demonstrated reduced constriction in response to carbachol.

Conclusions: These data demonstrate that the extracellular matrix protein mindin modifies the airway response to both LPS and ozone. Our data support a conserved role of mindin in production of proinflammatory cytokines and the development of AHR in two divergent models of reactive airways disease, as well as a role of mindin in airway smooth muscle contractility after exposure to ozone.

The article "The Role of the Extracellular Matrix Protein Mindin in Airway Response to Environmental Airways Injury" was retracted in 2016. Reasons: results that could not be reproduced; concerns about the data.

Asthma is a common disorder affecting 7–11% of the U.S. and European populations and is associated with substantial morbidity and health care costs (Bell et al. 2004; Dockery et al. 1993; Gryparis et al. 2004; Katsouyanni et al. 1995). The severity of asthma can be worsened by inhalation of commonly encountered environmental toxicants, including bacterial endotoxin and ambient air pollutants. Activation of innate immunity, in turn, can contribute to exacerbations of reactive airways disease. We previously reported the role of a prototypic gene of innate immunity, toll-like receptor 4 (*Tlr4*), in mediating the airway response to exposures to the environmental toxicants aerosolized lipopolysaccharide (LPS) and ozone (Hollingsworth et al. 2004).

LPS, also known as endotoxin, is found on the cell membranes of gram-negative bacteria and induces inflammation. LPS is ubiquitous in the environment. Experimental data from both mice (Schwartz 1996; Schwartz et al. 1994) and humans (Jagielo et al. 1996; O’Grady et al. 2001) show that LPS can cause airway obstruction that lasts as long as 48 hr immediately after a single exposure (Kline et al. 2000). Tlr4 is the transmembrane surface receptor for bacterial LPS. However, many genes likely can modify the response to inhaled endotoxin. We hypothesized that the gene mindin (spondin 2, extracellular matrix protein; *Spon2*) may contribute to the development of environmental airways disease. Mindin is an extracellular protein that contributes to pulmonary innate immune response (He et al. 2004) and allergic airways disease (Li H et al. 2006; Li Z et al. 2009).

Prior studies have demonstrated that, similar to Tlr4 (Hoshino et al. 1999; Poltorak et al. 1998), mindin is necessary for the biological response to LPS (He et al. 2004). For example, mindin regulates macrophage-dependent inflammatory response to LPS. Additionally, mindin contributes to integrin-dependent migration of macrophages (He et al. 2004; Jia et al. 2005). Therefore, deciphering a potential role for mindin in airway response to inhaled LPS would provide insight into mechanisms and establish more completely the innate immune response to LPS.

Increasing evidence supports the role of innate immunity in environmental airways disease. We now recognize that an endogenous ligand of surface receptor Tlr4 contributes to the biological response to ambient ozone (Garantziotis et al. 2009, 2010). Understanding the mechanisms that regulate the response to ambient ozone is of considerable interest to human health. Inhalation of ozone has been shown to contribute to increased morbidity and mortality in human populations (Bell et al. 2004; Gryparis et al. 2004; Ito et al. 2005; Levy et al. 2005; Parodi et al. 2005). Clear understanding of the host factors that contribute to the response to ozone is important for several reasons, including identification of susceptible individuals and the potential development of novel therapeutic interventions in reactive airways disease. Previous work supports that both mice (Kleeberger et al. 1997, 2000) and humans (Balmes et al. 1996; Weinmann et al. 1995a, 1995b) exhibit varying biological responses to ozone exposure, indicating that susceptibility to this toxicant may have a genetic basis. Genetic approaches to understanding the mechanisms that regulate response to ozone have highlighted the role of innate immunity. For example, previous studies support the role of innate immune proinflammatory factors in the biological response to inhaled ozone, including tumor necrosis factor-α (TNFα) (Cho et al. 2001; Kleeberger et al. 1997; Shore et al. 2001; Yang et al. 2005), interleukin (IL)-1β (Park et al. 2004), IL-6 (Johnston et al. 2005b), and KC (cytokine-induced neutrophil chemoattractant) (Driscoll et al. 1993; Johnston et al. 2005b). Cumulatively, these data support a role for innate immunity in the response to ambient ozone. However, the extracellular factors that contribute to the complete innate immune response to ambient ozone remain poorly understood.

The article "The Role of the Extracellular Matrix Protein Mindin in Airway Response to Environmental Airways Injury" was retracted in 2016. Reasons: results that could not be reproduced; concerns about the data.

The role of mindin in nonallergic airways disease has not previously been studied. Therefore, the goal of the present study was to determine the role of mindin in environmental airway injury to both inhaled LPS and ambient ozone using a mouse model. Our *in vivo* approach demonstrated that mindin was necessary for the complete response to both inhaled endotoxin and ambient ozone. Our observations build on the growing body of evidence supporting a fundamental role of the innate immune system in host response to noninfectious injury. We report that mindin-deficient (mindin^–/–^) mice have attenuated proinflammatory cytokine response and airway hyperresponsiveness (AHR) to both inhaled endotoxin and ambient ozone. These results support an essential role of mindin in host response to both of these models of airways disease and highlight the potential importance of host factors that modulate the complete innate immune response to commonly encountered environmental toxins.

## Materials and Methods

*Inbred mice.* C57BL/6J mice were purchased from Jackson Laboratory (Bar Harbor, ME). Mindin^–/–^ mice on a C57BL/6J background were generated as previously reported (He et al. 2004). All experimental protocols were reviewed and approved by the Institutional Animal Care and Use Committee at Duke University Medical Center and performed in accordance with the National Institutes of Health guidelines (Institute for Laboratory Animal Research 1996). Animals were treated humanely and with regard for alleviation of suffering. Each experimental group consisted of four or five male mice 6–8 weeks of age.

The article "The Role of the Extracellular Matrix Protein Mindin in Airway Response to Environmental Airways Injury" was retracted in 2016. Reasons: results that could not be reproduced; concerns about the data.

*Inhaled LPS protocol.* Animals were challenged with aerosolized LPS purified from 0111:B4 *Escherichia coli* (Sigma Aldrich, St. Louis, MO) for 2.5 hr. All animals were evaluated 4–7 hr after the initiation of LPS exposure. LPS at 0.9 μg/m^3^ in phosphate-buffered saline (PBS) was placed in a TSI jet nebulizer in a 55-L Hinners-style exposure chamber as previously reported (Hollingsworth et al. 2004). The dosage is similar to that experienced by workers in grain mills, swine confinement facilities, and the textile industry during a typical 8-hr work day and results in an inflammatory response in the lower respiratory tract (Simpson et al. 1999). C57BL/6J and mindin^–/–^ mice were exposed to either inhaled LPS or control saline solution (PBS). Data presented are representative of three individual experiments.

*Ozone protocol.* Animals were placed into separate caging and exposed in a chamber to filtered air (FA) or 1 ppm ozone for 3 hr and then allowed to recover for 24 hr under normal housing conditions. The level of ozone exposure (1 ppm for 3 hr) used in this protocol produced a minimum lung injury in terms of total and inflammatory cell counts in bronchoalveolar lavage fluid (BALF) compared with the more typical murine ozone injury model (2 ppm for 3 hr). Our selection of ozone concentration levels was based on similar biological responses observed in human exposure studies and published deposition fraction data for ozone in rodent models (Hatch et al. 1994; Wiester et al. 1988). This dose of ozone in mice is used to model the level of ozone encountered by humans during a “red” cautionary day as determined by the U.S. Environmental Protection Agency during the summer in many urban U.S. environments. Animals were exposed in the chamber with air at 20–22°C and 50–60% relative humidity supplied at a rate of 20 exchanges per hour. Ozone generated by directing 100% oxygen through an ultraviolet (UV) ozone generator was supplied after mixing with FA. The concentration of ozone in the exposure chamber was monitored continuously by an ozone UV light photometer (model 400E; Teledyne Technologies Inc., Thousand Oaks, CA). C57BL/6 and mindin^–/–^ mice were exposed to either ozone (1.0 ppm for 3 hr) or FA. Data presented are representative of three individual experiments.

The article "The Role of the Extracellular Matrix Protein Mindin in Airway Response to Environmental Airways Injury" was retracted in 2016. Reasons: results that could not be reproduced; concerns about the data.

*Lung lavage, cell counts, and analysis of supernatant.* As previously described by Garantziotis et al. (2009), mice were euthanized with CO_2_, and the lungs were exposed and fully inflated three times serially to 25 cm H_2_O with 0.9% NaCl. Cell counts were performed using a hemocytometer, and differentials were performed using hematoxylin and eosin–stained cytospins. Cell-free lavage supernatants were stored at –70°C. Cytokine/chemokines IL-1β, KC, MCP-1 (monocyte chemotactic protein-1), and TNF-α were determined by Luminex (Bio-Rad, Hercules, CA) using 5-plex reagents from Millipore (Billerica, MA). Assay sensitivities are 2.0 pg/mL for IL-1β, 1.4 pg/mL for KC, 5.3 pg/mL for MCP-1, and 1.0 pg/mL for TNF-α. Total protein concentrations in lung lavage fluid were measured by the Lowry Assay (Bio-Rad).

*AHR analysis.* Anesthesia was achieved with 60 mg/kg of pentobarbital sodium injected intraperitoneally. Mice were then given neuromuscular blockade (0.8 mL/kg pancuronium bromide) and ventilated with a computer-controlled small animal ventilator (FlexiVent; SCIREQ, Montreal, Quebec, Canada), with a tidal volume of 7.5 mL/kg  and a positive end-expiratory pressure of 3 cm H_2_O. Measurements of respiratory mechanics were made by the forced oscillation technique. Response to aerosolized methacholine (0, 10, 25, and 100 mg/mL) was determined by resistance measurements every 30 sec for 5 min, ensuring that the parameters calculated had peaked. The lungs were inflated to total lung capacity after each dose of methacholine, maintaining open airways and returning the measurements back to baseline. The resistance measurements were then averaged at each dose (R_T_, measured in centimeters of water per milliliter per second) along with the initial baseline measurement.

*Bronchial ring protocol.* Two bronchial rings from each mouse were studied simultaneously for their contractile response, as previously described (Du et al. 2005). Each bronchial ring was mounted horizontally on two tungsten triangles and submerged in modified Krebs buffer (118 mM NaCl, 4.8 mM KCl, 1.2 mM MgSO_4_, 1.2 mM KH_2_PO_4_, 2.5 mM CaCl_2_, 25 mM NaHCO_3_, 11 mM glucose; pH 7.4) in a thermostated organ bath constantly bubbled with a premixed gas consisting of 20% O_2_, 5% CO_2_, and balanced N_2_ at a constant temperature of 37°C. An optimal resting tension of 0.2 g was applied to each ring during the initial equilibration period of 30 min; the bronchial rings were then constricted with 80 mM KCl for 20 min to establish references for comparison. After washing off the excess KCl, the bronchial rings were treated stepwise with 100 nM to 3 μM (cumulative doses) carbachol at 5-min intervals, which allowed the contractile responses (isometric tensions) of bronchial rings to reach steady state after each carbachol dose. The increases in steady-state isometric tension of each bronchial ring caused by each carbachol dose were normalized against the length of the ring.

The article "The Role of the Extracellular Matrix Protein Mindin in Airway Response to Environmental Airways Injury" was retracted in 2016. Reasons: results that could not be reproduced; concerns about the data.

*Statistical analysis.* Data are expressed as mean ± SE. Significant differences between groups were identified by analysis of variance, and individual comparisons are made using unpaired two-tailed Student *t*-tests. A *p*-value < 0.05 was considered statistically significant.

## Results

*Mindin-dependent response to inhaled LPS.* We first investigated whether the absence of mindin affects the airway response to methacholine in control mice after exposure to saline aerosol. At 4–7 hr postexposure, we observed no detectable differences induced by saline in a mindin-dependent manner (Figure 1A). However, after exposure to LPS, C57BL/6J mice exhibited significantly higher airway responsiveness than did mindin^–/–^ mice. Similarly, we found a significant difference between saline-challenged mindin^–/–^ mice and LPS-exposed mindin^–/–^ mice. The LPS-challenged mindin^–/–^ mice exhibited significantly lower airway responsiveness than did LPS-challenged C57BL/6J mice (Figure 1B).

**Figure 1:** Airway responsiveness in C57BL/6J and mindin^–/–^ mice before (*A*) and after (*B*) challenge with inhaled LPS (*n* = 5/group). Baseline values with methacholine challenge were similar in unexposed animals (*A*); however, after LPS exposure (*B*), C57BL/6J mice showed significantly increased airway responsiveness compared with LPS-exposed mindin^–/–^ mice. *p < 0.05.

Next, we characterized cellular recruitment into the airspace in C57BL/6J and mindin^–/–^ mice exposed to either saline or LPS. LPS exposure in both C57BL/6J and mindin^–/–^ mice resulted in an increase in total cells and a higher absolute number of neutrophils in whole-lung lavage fluid compared with saline (Figure 2A). However, LPS-exposed mindin^–/–^ mice demonstrated significantly fewer total cells and neutrophils compared with LPS-exposed C57BL/6J mice (Figure 2B).

**Figure 2:** Cellular recruitment into the airspace (*A,B*) and total protein level (*C*) measured in whole-lung lavage fluid from C57BL/6J and mindin^–/–^ mice after exposure to saline or LPS (*n* = 5/group). Cellular recruitment into the airspace was evaluated by the number of total cells (*A*) and the number of neutrophils (*B*). Mindin^–/–^ mice demonstrate reduced cellular inflammation after exposure to LPS compared with C57BL/6J mice. Mindin^–/–^ mice do not have a detectable increase in total protein after exposure to LPS (*C*). *p < 0.05 for LPS-exposed C57BL/6J mice compared with either group of saline controls. **p < 0.05 for LPS-exposed C57BL/6J mice compared with LPS-exposed mindin^–/–^ mice.

The article "The Role of the Extracellular Matrix Protein Mindin in Airway Response to Environmental Airways Injury" was retracted in 2016. Reasons: results that could not be reproduced; concerns about the data.

Total protein in whole-lung lavage fluid indicates epithelial permeability or lung injury. After exposure to LPS, C57BL/6J mice demonstrated significantly higher levels of total protein in whole lung lavage fluid compared with saline-challenged genetic counterparts (Figure 2C). In contrast, we found no significant difference between LPS-exposed mindin^–/–^ mice and their saline-exposed counterparts (Figure 2C). We observed a trend toward reduced level of total protein after exposure to LPS in mindin^–/–^ mice compared with C57BL/6J mice (*p* = 0.07).

We measured the level of nuclear factor κB–dependent cytokines in the BALF as a marker of activation of innate immunity. After LPS exposure, C57BL/6J mice had notable increases in KC, IL-1β, MCP-1, and TNF-α in BALF compared with saline-exposed mice (Figure 3). Cytokines in LPS-exposed mindin^–/–^ mice were also increased compared with saline counterparts, but cytokines were significantly reduced compared with LPS-exposed C57BL/6J mice (Figure 3).

**Figure 3:** Proinflammatory cytokines KC (*A*), IL-1β (*B*), MCP-1 (*C*), and TNF-α (*D*) measured in BALF from C57BL/6J and mindin^–/–^ mice after exposure to saline or LPS (*n* = 5/group). *p < 0.05 for LPS-exposed C57BL/6J mice compared with either group of saline controls. **p < 0.05 for LPS-exposed C57BL/6J mice compared with LPS-exposed mindin^–/–^ mice.

*Mindin-dependent response to inhaled ozone.* To determine whether mindin contributes to airway response after inhaled ozone, we challenged mice acutely with either FA or ozone (1 ppm for 3 hr), and at 20–24 hr postexposure we characterized them for airway sensitivity to methacholine challenge. We observed no baseline differences between C57BL/6J and mindin^–/–^ mice in methacholine sensitivity after exposure to FA (Figure 4A). As anticipated, we found a significant difference in AHR in C57BL/6J mice exposed to FA and ozone (Figure 4B). However, mindin^–/–^ mice showed no significant differences in sensitivity to methacholine between FA-exposed and ozone-exposed mice. Thus, mindin^–/–^ mice exhibited a significant reduction in AHR after ozone compared with C57BL/6J mice.

**Figure 4:** Airway responsiveness in C57BL/6J and mindin^–/–^ mice before (*n* = 4/group; *A*) and after (*n* = 5/group; *B*) challenge with ozone. *p < 0.05 compared with ozone-exposed mindin^–/–^ mice.

We also characterized cellular recruitment into the airspace at 20–24 hr after ozone exposure. We found increased numbers of total cells and neutrophils after inhalation in both strains of mice, but there were no significant differences in total cells or neutrophils by genotype (Figure 5A,B).

The article "The Role of the Extracellular Matrix Protein Mindin in Airway Response to Environmental Airways Injury" was retracted in 2016. Reasons: results that could not be reproduced; concerns about the data.

**Figure 5:** Cellular recruitment into the airspace, evaluated by the number of total cells (*A*) and the number of neutrophils (*B*), and total protein level (*C*) measured in whole-lung lavage fluid from C57BL/6J and mindin^–/–^ mice after exposure to FA or ozone (*n* = 5 per group). *p < 0.05 for ozone-exposed C57BL/6J mice compared with either group of FA-exposed controls. ^#^*p* < 0.05 for ozone-exposed mindin^–/–^ mice compared with either group of FA-exposed controls.

The total protein assays yielded a significant difference in BALF total protein between ozone-exposed wild-type mice and their FA-exposed counterparts (Figure 5C). After exposure to ozone, both the C57BL/6J and mindin^–/–^ mice exhibited higher levels of total protein in whole-lung lavage fluid. The level of BALF total protein in response to ozone appears to be independent of mindin.

To determine activation of innate immunity, we measured levels of specific proinflammatory cytokines previously associated with ozone-induced AHR. As anticipated, ozone-exposed C57BL/6J mice had significantly higher concentrations of KC, IL-1β, MCP-1, and TNF-α compared with FA-exposed C57BL/6J mice. In ozone-exposed mindin^–/–^ mice, the concentrations of these proinflammatory cytokines were increased compared with FA controls. However, inflammatory cytokine levels in BALF collected from the mindin^–/–^ mice were significantly decreased compared with those from ozone-exposed C57BL/6J mice (Figure 6).

**Figure 6:** Proinflammatory cytokines KC (*A*), IL-1β (*B*), MCP-1 (*C*), and TNF-α (*D*) measured in the BALF from C57BL/6 and mindin^–/–^ mice after exposure to FA or ozone (*n* = 5/group). *p < 0.05 for ozone-exposed C57BL/6J mice compared with either group of FA-exposed controls. **p < 0.05 for ozone-exposed C57BL/6J mice compared with ozone-exposed mindin^–/–^ mice.

*Mindin-dependent bronchial ring contractility.* To determine whether mindin contributes to airway smooth muscle contractility, we examined bronchial ring contractile response to carbachol. We observed no baseline differences in bronchial ring contractile response in unexposed (Figure 7A) or LPS-exposed mindin^–/–^ or C57BL/6J mice (Figure 7B). However, we did observe significant mindin-dependent differences in bronchial ring contractility to carbachol 24 hr after inhalation of ozone (Figure 7C), in agreement with previous data suggesting that inhalation of ozone may enhance airway smooth muscle contraction (Yoshida et al. 2002). Together, these observations support that mindin contributes to airway smooth muscle contractility after inhalation of ozone but not at baseline or after inhalation of LPS.

The article "The Role of the Extracellular Matrix Protein Mindin in Airway Response to Environmental Airways Injury" was retracted in 2016. Reasons: results that could not be reproduced; concerns about the data.

**Figure 7:** Bronchial ring contractile response to carbachol in naive (*A*), LPS-exposed (*B*), and ozone-exposed (*C*) C57BL/6J and mindin^–/– ^mice.**In *A*, *n* = 6 for C57BL/6J and *n* = 5 for mindin^–/–^; in *B*, *n* = 6 for C57BL/6J and *n* = 6 for mindin^–/–^; in *C*, *n* = 9 for C57BL/6J and *n* = 8 for mindin^–/–^. *p < 0.05 for ozone-exposed C57BL/6J mice compared with ozone-exposed mindin^–/–^ mice.

## Discussion

Our findings support the conclusion that mindin plays a modifying role in innate immune response to the inhaled toxicants endotoxin and ozone. We demonstrate that mindin^–/–^ mice have divergent degrees of protection from the biological response to either inhaled LPS or ozone. Specifically, mindin^–/–^mice have attenuation of AHR and proinflammatory cytokines in response to both endotoxin and ozone. These observations are strikingly similar to AHR and inflammatory phenotypes previously observed in the Tlr4^–/–^ mouse (Hollingsworth et al. 2004). Collectively, these observations suggest that mindin contributes to activation of innate immunity in the context of environmental airways injury. Our observations further highlight the importance of genes that modify innate immunity in reactive airways disease and response to commonly encountered inhaled environmental toxicants.

The apparent similarities between Tlr4^–/–^ mice and mindin^–/–^ mice in responses to LPS and ozone are quite remarkable. We previously observed complete protection in the Tlr4^–/–^ mouse (Hollingsworth et al. 2004), whereas in the present study we saw an attenuated response to LPS and ozone in the mindin^–/–^ mouse, despite similar levels of *Tlr4* mRNA expression in whole lung [see Supplemental Material, Figure 1A,B (http://dx.doi.org/10.1289/ehp.1003339)]. This finding suggests that mindin functions as a modifier gene in response to endotoxin, an observation consistent with our current understanding that mindin is located in the extracellular compartment and facilitates interaction between the carbohydrate domain of LPS with the Tlr4 surface receptor (He et al. 2004). It is equally intriguing that both the Tlr4-dependent and mindin-dependent responses to ozone similarly affect only the profile of proinflammatory cytokines and the development of AHR. After exposure to ozone, total BALF protein is largely independent of either Tlr4 or mindin (Hollingsworth et al. 2004).This observation suggests that changes in permeability or lung injury are generally independent of these genes of innate immunity in these models of environmental lung injury.

The article "The Role of the Extracellular Matrix Protein Mindin in Airway Response to Environmental Airways Injury" was retracted in 2016. Reasons: results that could not be reproduced; concerns about the data.

Although we observed differences in mRNA expression of mindin in whole lung after exposure to LPS [see Supplemental Material, Figure 1C (http://dx.doi.org/10.1289/ehp.1003339)], we observed no such differences after inhalation of ozone (see Supplemental Material, Figure 1D). It is therefore plausible that either the level of mindin expression or posttranslational modifications of extracellular mindin could contribute to interaction with Tlr4 surface recognition. However, the specific mechanism by which mindin contributes to the response to ozone remains unknown and will be a focus of future investigations.

Previous work supports that mindin, as part of the extracellular matrix, provides a lattice required for integrin-dependent binding and recruitment of inflammatory cells, including macrophages, neutrophils (Jia et al. 2005), and eosinophils (Li et al. 2009). Mindin contributed to reactive airways disease in the ovalbumin model, which was associated with a defect in eosinophil recruitment (Li et al. 2009). It remains unclear whether the mindin-dependent differences in AHR in the allergic model of reactive airways disease are indirectly related to observed differences in granulocyte recruitment. We consistently observed that mindin^–/–^ mice exposed to LPS had impaired recruitment of inflammatory cells to the lung. Thus, mindin-dependent differences in AHR after exposure to LPS are associated with defects in inflammatory cell recruitment. From this standpoint, our results regarding ozone exposure may provide additional insight into the biological role of mindin. After ozone, recruitment of inflammatory cells to the airspace was mindin independent, yet we observed mindin-dependent defects in both inflammatory cytokines and AHR. This observation suggests that the mechanisms that contribute to ozone-induced AHR are independent of cellular inflammation. We previously observed that direct instillation of hyaluronan fragments into the lung can induce AHR in a manner independent of cellular inflammation (Garantziotis et al. 2009). Therefore, we considered that because mindin binding to LPS can be blocked by simple sugars (He et al. 2004), mindin could be required for biological response to hyaluronan fragments, which contribute to Tlr4-dependent response to ozone (Garantziotis et al. 2009, 2010). However, we determined that the *in vivo* AHR response to hyaluronan fragments in the airspace is independent of mindin [see Supplemental Material, Figure 2 (http://dx.doi.org/10.1289/ehp.1003339)]. Next, we considered the possibility that mindin directly contributes to airway smooth muscle contractility. Although we did not observe mindin-dependent differences in carbachol-induced contraction of bronchial rings in either unexposed or LPS-exposed mice, we were surprised to find that mindin^–/–^ mice were protected from carbachol-induced bronchial ring contraction after inhalation of ozone (Figure 7). This finding is quite interesting for two reasons: First, very little is known about the impact of ozone inhalation on airway smooth muscle contractility, and second, we identified a novel role for mindin in airway smooth muscle function. However, the specific mechanism by which mindin can modify airway smooth muscle contractility after inhalation of ozone remains unknown and will be an area of future investigation.

The article "The Role of the Extracellular Matrix Protein Mindin in Airway Response to Environmental Airways Injury" was retracted in 2016. Reasons: results that could not be reproduced; concerns about the data.

Our results in the ozone model of AHR support a direct role of innate immune activation in the severity of reactive airways disease. For this reason, we consider the possible therapeutic implications of inhibition of pulmonary innate immunity during exacerbations of existing airways disease. Intensity of innate immune response is a double-edged sword—precise regulation is required to optimize both normal inflammation and resolution of tissue injury. It appears that the intensity of innate immune activation can produce divergent effects on the host. For example, low-level Tlr4 signaling appears protective in some forms of oxidative lung injury (Qureshi et al. 2006; Zhang et al. 2005, 2006), moderate Tlr4 signaling facilitates the clearance of pathogens (Chassin et al. 2009; Wieland et al. 2005), and excessive prolonged Tlr4 signaling can augment lung injury (Brass et al. 2008). The future challenge of therapeutic development will be controlled attenuation of excessive and prolonged proinflammatory response without impairing intact host antibacterial defense. Understanding the basic mechanisms that regulate host innate immune response to both infectious and noninfectious lung injuries can provide the insight required for successful therapeutic development. Previous work supports that both Tlr4 and mindin play a fundamental role in antibacterial host defense. It is unclear if targeting the extracellular matrix protein mindin and/or Tlr4 receptors in airway disease with an AHR clinical phenotype would provide significant clinical benefit. However, a clearer understanding of host factors in response to common environmental exposures can provide insight for the future development of personalized therapies with a basis in pharmacogenetics.

## Conclusions

The extracellular matrix protein mindin is an important modifier of pulmonary innate immune response to commonly inhaled environmental toxicants. Mindin plays a central role in the biological response to both inhaled LPS and ambient ozone. Mindin^–/–^ mice demonstrated reduced AHR and production of proinflammatory cytokines in these two divergent models of environmental airways injury. Mindin contributed to bronchial ring contractility only after inhalation of ozone. Clear understanding of the mechanisms that mindin contributes to the development of reactive airways disease could provide an opportunity for development of novel therapeutic strategies in human reactive airways disease.

The article "The Role of the Extracellular Matrix Protein Mindin in Airway Response to Environmental Airways Injury" was retracted in 2016. Reasons: results that could not be reproduced; concerns about the data.

## Supplemental Material

(88 KB) PDF
